The article "Recent Trends of Polymer Mediated Liposomal Gene Delivery System" was retracted in 2019. Reasons: plagiarized text; overlap with other authors' work.

# Recent Trends of Polymer Mediated Liposomal Gene Delivery System

**DOI:** 10.1155/2014/934605

**Published:** 2014-08-27

**Authors:** Shyamal Kumar Kundu, Ashish Ranjan Sharma, Sang-Soo Lee, Garima Sharma, C. George Priya Doss, Shin Yagihara, Do-Young Kim, Ju-Suk Nam, Chiranjib Chakraborty

**Affiliations:** ^1^Department of Physics, School of Basic and Applied Sciences, Galgotias University, Greater Noida 203201, India; ^2^Department of Physics, Tokai University, Hiratsuka-Shi, Kanagawa 259-1292, Japan; ^3^Institute for Skeletal Aging & Orthopedic Surgery, Hallym University-Chuncheon Sacred Heart Hospital, Chuncheon 200704, Republic of Korea; ^4^Medical Biotechnology Division, School of Biosciences and Technology, VIT University, Vellore, Tamil Nadu 632014, India; ^5^Department of Bioinformatics, School of Computer Sciences, Galgotias University, Greater Noida 203201, India

## Abstract

Advancement in the gene delivery system have resulted in clinical successes in gene therapy for patients with several genetic diseases, such as immunodeficiency diseases, X-linked adrenoleukodystrophy (X-ALD) blindness, thalassemia, and many more. Among various delivery systems, liposomal mediated gene delivery route is offering great promises for gene therapy. This review is an attempt to depict a portrait about the polymer based liposomal gene delivery systems and their future applications. Herein, we have discussed in detail the characteristics of liposome, importance of polymer for liposome formulation, gene delivery, and future direction of liposome based gene delivery as a whole.

## 1. Introduction

The gene therapy has shown great promise for the potential cure of several genetic disorders and appears to possess enormous therapeutic potential. Although this news might seem fresh and innovative, the transfer of genetic materials into living cells has been tested around the decades. In 1966, Tatum [1] predicted that the transfection techniques for mammalian cells will be advertised as part of the future medicine. After over 30 years of research, the field of gene therapy is offering an acceptable treatment protocol for the cure for human diseases.

Studying the basic structure of genes into cells of different origins has been a major practice in cellular biology investigation. In addition to being a powerful research implement, gene transfer is a novel idea for gene therapy and is a molecular therapeutic approach for curing inherited and several other diseases [2, 3]. Diseases developed because of a genetic constituent can theoretically be corrected by genetic refinement based on the addition of needed genes. Among the genetic diseases, muscular dystrophy, cystic fibrosis, and familial hypercholesteremia have been studied so far. As for cancer, most of the mutations acquired are not inherited but are a result of cumulative effect of various external factors. Therefore, it is a great challenge in the area of gene therapy to correct these mutations and to repair the gene. A gene itself is not able to enter into a cell as it is a large portion of DNA that is bound by several anionic charges. A wide range of artificial techniques has been developed and utilized time to time for* in vitro* gene transfer. Some techniques of gene transfer are membrane perturbation by chemicals (i.e., organic solvents and detergents), direct DNA microinjection, physical methods (i.e., mechanical or osmotic method and electric shocks), and liposomes.

The article "Recent Trends of Polymer Mediated Liposomal Gene Delivery System" was retracted in 2019. Reasons: plagiarized text; overlap with other authors' work.

Intent of gene delivery approaches is to introduce genetic material into patients' cells. Subsequent successful gene transfer in these cells will produce a therapeutic protein that will counter the cause of disease. However, the safety apprehensions and the difficulties related to production on large scale are the drawbacks that are associated with recombinant viral vectors [4] which has prompted the search for efficient, nonimmunogenic, and easy to prepare nonviral vector systems. The effectiveness of amounts of drugs is often restricted by their potential to reach the site of therapeutic effect. In many cases, the majority of drugs allocate all over the body with its physicochemical and biochemical properties while only a minor amount of a controlled dose reaches the targeted area. Therefore, emerging drug delivery system enhances the pharmaceutical effect of drugs while reducing its toxicity* in vivo* which is a challenging task. Lipid molecules of  biomembranes interacting with water molecules can control the transport phenomena and protein functions with anisotropic flow ability. For formulating lipid-based drug carrier systems, a consistent and repeatable exploration of their size, as well as size allocation, is of paramount importance for the nanocarrier's* in-vitro* characteristics for example, drug loading capacity, aggregation, sedimentation, and so forth [5, 6]. A considerable attention has been paid for liposomal drug delivery systems owing to their specific attractions, that is, (1) fruitful encapsulation of together tiny and large molecules (e.g., antigens) with a wide range of hydrophobic levels and pKa values, (2) prolonging and target release of therapeutic molecule/agent by alteration of liposome surface, and (3) minimization of clinical drug dose and reducing toxicity effects [7, 8].

Improvements in lipofection technique by surface modifications with polyethylene glycol (PEG) have facilitated the safety from degradation* in vivo*. Surface amendment of drug delivery systems with PEG has encountered increasing interest to enhance biocompatibility [9], increase in systemic circulation times [10], and change in their biodistribution [11]. For example, nanoparticles [12], liposomes [13], and also adenoviruses [14] have been “PEGylated” mainly to obtain long-circulating particulate delivery systems, based on the “stealth” effect. In the year 2002, Bhadra et al. [15] reviewed the PEGylation methodology. PEGylation of polycations for the purpose of gene delivery has been realized to block and graft copolymers [16, 17]. PEG offers numerous attractive potential as a liposomal covering and is obtainable in wide variety of molecular weights. Due to lack of toxicity, it is excreted easily by the kidneys and also eases for application purpose [18]. Modifications of liposomal surfaces with PEG are achieved either by its physical adsorption onto the liposomal surface or its covalent attachment onto premade liposomes [19].

The article "Recent Trends of Polymer Mediated Liposomal Gene Delivery System" was retracted in 2019. Reasons: plagiarized text; overlap with other authors' work.

The primary objective of this review article is to describe the polymer based liposomal gene delivery system and its potential applications. To achieve this objective, we have illustrated the topics in several headings such as characteristics of liposome, importance of polymer for liposome formulation, gene delivery, and future direction of liposome-based gene delivery.

## 2. Characteristics of Liposome

Innovative studies using liposomes were first performed by Bangham et al. roughly 50 years ago. [20–22]. From these studies, it was recognized that phospholipids in aqueous systems are made up of closed bilayer structures. Liposomes have passed through several practical applications to become pharmaceutical carrier of choice from just another exotic object of biophysical research. The real breakthroughs in this area were established during the past 20 years, which witnessed approval of many liposomal drugs as well as the presence of different unique biomedical products in pharmaceutical sector. Presently, several types of liposomes are available for gene delivery system. Therefore, the development of the technologies for the liposome delivery systems is an exciting area having both, clinical and economic values.

### 2.1. Liposomes Can Be Produced by the Self-Assembly

In general, liposomes are formed by the self-assembly of dissolved lipid molecules. Lipid molecules contain a hydrophilic head group and hydrophobic tails. These lipid molecules form an association which yields entropically favorable states of lower free energy and in some cases appear to form bimolecular lipid leaflets. Such leaflets are categorized by hydrophobic hydrocarbon tails facing each other to avoid water molecules and hydrophilic head groups pointing outward to associate with water molecules [23]. At this an argument exists that the bilayer formation is still energetically unfavorable as the hydrophobic portion of the molecules is still in contact with water. This difficulty has been solved by forming a vesicle with closed edges through the curvature of developing bilayer membrane upon itself [24]. Therefore, the free-energy-driven self-assembly is steady and has been exploited as powerful machinery for liposomes for a particular given system [25].

The article "Recent Trends of Polymer Mediated Liposomal Gene Delivery System" was retracted in 2019. Reasons: plagiarized text; overlap with other authors' work.

### 2.2. Liposomes Are Spherical, Self-Assembling Vesicles with One or Several Lipid Bilayers

Liposomes are spherical, self-assembling vesicles formed by one or several lipid bilayers leaving an aqueous core inside. The lipid bilayers are composed of amphiphilic lipids, derived from or based on the structure of biological membrane lipids. The hydrophobic part of the lipid is designed of two hydrocarbon chains, which naturally vary from 8 to 18 carbons in length, and it can be either saturated or nonsaturated. A membrane with a gel phase (L_*β*_) is made by long and saturated acyl chains resulting in increased stability and rigidity of the liposomes. On the other hand, the use of short and/or unsaturated acyl chains results in more fluid, liquid crystalline (L_α_) bilayer structure. Experimentally, this gel-liquid crystal (LC) phase transition is well observed by changing temperature [26, 27]. Addition of cholesterol into the lipid bilayer minimizes the effects of membrane permeability and improves the mechanical strength of the liposomes. Surface charge of the liposome can be affected strongly by varying the hydrophilic head group of the lipid which are either zwitterionic [e.g., phosphatidylcholine (PC) and phosphatidylethanolamine (PE)], negatively charged [e.g., phosphatidylglycerol (PG)], or positively charged [e.g., 3-trimethylammonium-propane (TAP)] [8]. In the water, amphiphilic lipids tend to form bilayer structure as they are poorly soluble in water with a critical micelle concentration (CMC).

### 2.3. Hydrophobic Drug Molecules Can Be Entrapped Easily through the Lipid Bilayer of Liposomes

Hydrophobic drug molecules can be entrapped passively in the lipid bilayer through the preparation of liposomes. Such drug molecules are encapsulated in the aqueous core of the liposome or the aqueous phase between bilayers (in the case of multilamellar vesicles) using passive loading methods, such as reverse phase evaporation [28], dehydration-rehydration method [29], or active loading involving pH-gradient across the liposome membrane [30, 31]. Remote filling of doxorubicin into preformed liposomes by means of ammonium sulfate gradient as a driving force results in the efficient and stable entrapment of the drug [32]. Some liposomal cancer drugs that are currently employed clinically utilise remote loading such as Caelyx and Myocet loaded with doxorubicin and Daunoxome with daunorubicin.

The article "Recent Trends of Polymer Mediated Liposomal Gene Delivery System" was retracted in 2019. Reasons: plagiarized text; overlap with other authors' work.

### 2.4. Liposome Delivery System Can Be Developed into a Variety of Sizes

Liposomes may exhibit a variety of sizes and morphologies contrary for the assembling of lipids or lipid blends suspended in an aqueous medium [33]. The unilamellar vesicle is a common morphology which is analogous to the eukaryotic cellular membrane. This vehicle is characterized by a single bilayer membrane that encapsulates an internal aqueous solution, therefore, separating it from the external (bulk) solution [34]. Both anionic phospholipid and cationic amine head groups are responsible for forming single-walled vesicles. Vesicle sizes are covered in the range of nanometer to micrometer. Spontaneously formed multilamellar vesicles (MLV) are very heterogeneous in lamellarity and size, ranging from 500 nm to 5 *μ*m. More sophisticated, small unilamellar vesicles (SUV, <100 nm) and large unilamellar vesicles (LUV, 100–800 nm) can be prepared by sonication or extrusion [27, 33, 35].

Giant or gigantic vesicles also comprise additional morphologies such as (i) multilamellar, which consists of many concentric bilayers, (ii) oligolamellar, which consists of only two concentric bilayers, and (iii) multivesicular, which consists of various smaller unilamellar vesicles inside of one giant one. With the exception of multilamellar vesicles, other morphologies are very difficult to obtain without highly controlled processes of creation [33]. Giant vesicles also have the merit of attention owing to their large sizes, ranging from 1 *μ*m to more than 100 *μ*m [33]. These large vesicles have been extensively studied and well characterized so far, partially due to ease of observation [36].

### 2.5. Liposome Assemblies

A number of assemblies have been recognized [37–42] during the compaction of polynucleotides into liposomal associations. Each of such structures is created in the utmost energetically favorable conformation, relying on the features of the definite lipids used in the system [43]. Here the structure-packing parameter can be used to recommend the possible shape of the amphiphile, which in turn depends on the ratio of size variables. The main drawbacks pertaining to the use of liposomes are the swift elimination from the blood and trapping of the lipid assemblies by the cells of the reticuloendothelial system, predominantly in the liver. A number of improvements are being tried to reduce this shortcomings of liposomes.

The article "Recent Trends of Polymer Mediated Liposomal Gene Delivery System" was retracted in 2019. Reasons: plagiarized text; overlap with other authors' work.

### 2.6. Liposome and Surface-Attached Ligands

It has been proposed that the use of targeted liposomes with surface-attached ligands, capable of recognizing and binding to cells of interest, may help in increasing liposomal drug accumulation in the desired tissues and organs. For example, immunoglobulins (Ig) of the IgG class and their fragments are extensively used in targeting moieties that can be attached to liposomes. Nothing has been found to affect the liposomal integrity or the antibody properties that are bound covalently to the liposome surface or by the hydrophobic interaction with the liposomal membrane after alteration with hydrophobic residues [44]. Nevertheless, despite improvements in the targeting efficacy, major proportion of immune-liposomes is found accumulated in the liver as a consequence of inadequate time for the communication between the target and targeted liposomes. Hence, a better target accumulation can only be achieved if liposomes are maintained for long circulation time in blood stream.

Different methods have been recommended for achieving long circulation of liposomes* in vivo*, including coating of the liposomal surface with inert, biocompatible polymers, such as PEG. PEG forms a protective layer over the liposomal surface and slows down the liposome recognition by opsonins [45, 46]. Long-circulating liposomes are being scrutinized in detail and are extensively used in biomedical* in vitro* and* in vivo* studies also leading their way into clinical practices [47, 48]. A significant role of protecting polymers is because of their flexibility which permits comparatively small number of surface-grafted polymers to create an impermeable layer above the liposome surface [49, 50]. Long-circulating liposomes exhibit dose-independent, nonsaturable, log-linear kinetics and increased bioavailability [51].

### 2.7. Liposome and Gene Delivery

The challenges being faced for the development of various techniques for liposomal gene delivery systems are not unlike compared to those that are being faced for liposomal drug delivery systems. The therapeutic listing of the conservative or gene-based drugs (e.g., plasmid DNA or RNA transcripts) are enhanced by delivering more biologically active drug to target cells or tissues, to circumvent drug-related toxicities. By means of gene-based drugs, the delivery into suitable cells denotes only a part of the problem. A number of intracellular barriers are present in many cell types that can inhibit the biologic activity of gene-based drugs [52, 53]. It is not very obvious what role, if any, liposomes will play in overcoming these intracellular barriers.

The article "Recent Trends of Polymer Mediated Liposomal Gene Delivery System" was retracted in 2019. Reasons: plagiarized text; overlap with other authors' work.

### 2.8. Liposome and DNA Delivery

The liposome based DNA delivery was recognized as early as late 1970s [54]. On the other hand, gene-based drugs have presented interesting challenges for systemic delivery systems. The gene-based drugs are highly susceptible to degradation by the nucleases present in plasma. Although liposomes have the potential to encapsulate gene-based drugs and prevent inactivation by nucleases, but methods used to encapsulate plasmid DNA efficiently are not well defined, small liposomes or lipidic DNA particles have only been appreciated. The usefulness of gene-based drugs is absolutely dependent on gaining entry into the target cell cytosol in an intact form. Consequently, for effectiveness of liposomes, they must act as integrate agents that endorse intracellular delivery. With a few exceptions (e.g., skeletal muscle [55, 56] such as hepatocytes [57, 58]), naked plasmid DNA alone is not taken up very efficiently by most of the cell types* in vivo*. For certain gene therapy approaches, such as those involving the delivery of suicide genes, systemic gene delivery systems must have the potential to deliver gene-based drugs selectively to specific target cells.

Drug loading capacity are achieved either actively (i.e., after liposome formation) or passively (i.e., the drug is encapsulated during liposome formation). Hydrophobic drugs are directly incorporated into liposomes through vesicle formation. The magnitude of uptake and retention is controlled by lipid-drug interactions. Trapping efficiency of 100% is frequently attainable but totally relies on the solubility of the drug in the liposome membrane. During vesicle formation, the passive encapsulation of water-soluble drugs depends on the capability of liposomes to hold aqueous buffer containing a drug suspension easily. Trapping efficiency is restricted (usually less than 30%) by the trapped volume confined in the liposomes and drug solubility. Additional method to enhance the passive encapsulation of water-soluble drugs is to give an amphipathic nature to the drugs by conjugating or complexing the drugs to lipids [59, 60]. Instead, water-soluble drugs that have ionizable amine functions are actively entrapped by employing pH gradients [61], which results in trapping efficiencies approaching 100%.

Cationic liposomes (lipoplexes) are the most frequently used in nonviral gene transfer systems. Nevertheless, in contact with negatively charged DNA, lipid molecules form electrostatic complexes with DNA. In the meantime, the pioneering work of Felgner and Ringold [62] introduced cationic DOTMA/DOPE liposomes and numerous other cationic lipids that have been designated. Selected lipids have monovalent head groups, for example, DOTMA [62] and DOTAP [63], and some others, like DOGS and DPPES [64], include multivalent head groups. Cationic lipids may also include a neutral fusogenic lipid, dioleoylphosphatidylethanolamine (DOPE). Complexes of cationic lipids with genes are heterogeneous [65, 66] and susceptible to changes in the surrounding solution [67]. Cationic liposomes have been studied* in vitro*,* in vivo*, and even in clinical trials [68], but the main difficulty that remains to be resolved is low transfection efficiency for* in vivo* applications. Although the endosomal buffering capacity has not been proven directly, but due to the p*K*_*a*_ values of their secondary and tertiary amines, it is widely believed [64, 69–72] that polyethyleneimines and dendrimers, as well as DOGS lipid, may buffer endosomes.

The article "Recent Trends of Polymer Mediated Liposomal Gene Delivery System" was retracted in 2019. Reasons: plagiarized text; overlap with other authors' work.

## 3. Importance of Polymer for Liposome Formulation

### 3.1. PEG-Liposomes and Their Uses in Different Diseases

Kim and his coworkers revealed that PEGylated lipoplexes yield amplified transfection efficiencies in the occurrence of serum as compared to liposomal transfection methods. The PEGylated lipoplexes presented enhanced stabilities and longer passage times in the blood. It is supposed that the PEG forms a steric barrier surrounding lipoplexes, which stifles clearance due to compact macrophagocytes uptake [19], and may permit the liposome to overcome accumulation problems over mutually repulsive interactions between PEG molecules [73]. These characteristics facilitate higher transfection efficiencies, increased bioavailability, due to larger available concentrations, and improved tissue distribution [74]. These particles are sometimes denoted as “stealth liposomes,” since they can decrease immune responses and improve circulation time associated with PEG-modified liposomes. By means of cellular targeting, such liposomes lack specificity. Shi et al. [75] developed the technique to inhibit the endocytosis through PEGylation of the lipoplexes that was dependent upon the mole fraction of PEG on the liposome. It has unique functional groups that are combined with the lipoplexes. PEG on the liposome is a proper complex, which separates DNA packing upon incorporation into the cell. Based on these findings, a need has arisen for the formation of PEG-containing liposomes, whereby the attached PEG is detached following endocytosis via a hydrolysable connecting molecule. Thus, current researches on PEG-liposomes are focused on joining the PEG in a removable fashion to facilitate liposome capture by the cells. The PEG coating is separated during the performance of some pathological conditions (decreased pH in tumours). It has been found that the enhanced permeability and retention (EPR) cause PEG-liposomes accumulation at the target site [76]. A new detachable PEG conjugates have been described by Zalipsky et al. [77], wherein the detachment process mainly depends on the mild thiolysis of the dithiobenzylurethane, linked between PEG and amino-containing substrates.

The article "Recent Trends of Polymer Mediated Liposomal Gene Delivery System" was retracted in 2019. Reasons: plagiarized text; overlap with other authors' work.

The delivery of the anticancer agent doxorubicin in PEG liposomes has been found for treatment of solid tumours with breast-carcinoma metastases patients, and it resulted in a subsequent improvement in survival [78–80]. The similar set of indications was targeted by a combination therapy comprising liposomal doxorubicin and paclitaxel [81] as well as Caelyx (Schering-Plough) (doxorubicin in PEG liposomes) and carboplatin [82]. For patients, the Caelyx is in Phase II clinical trials with squamous cell cancer of the head and neck [83] and ovarian cancer [84]. Clinical research revealed that the effect of doxorubicin in PEG liposomes is very impressive against unresectable hepatocellular carcinoma [85], cutaneous T-cell lymphoma [86], and sarcoma [87]. Liposomal lurtotecan was presented to be effective in patients with topotecan-resistant ovarian cancer [88]. Additional signs targeted by liposomal formulations include amphotericin B for the treatment of visceral leishmaniasis [89] and liposomal bupivacaine long-acting analgesia [90].

### 3.2. PEG Co-Polymers and Its Assembly

Among various strategies to provide elements with stealth-shielding, incorporate surface modification with poly(acrylamide), poly(vinyl alcohol), and polysaccharides as well as surface modification with PEG and PEG copolymers was found to be the most effective methods. Wide-spread use of those elements was noted in these references [91–93]. PEG has a universal assembly of HO–(CH_2_CH_2_O)_*n*_–CH_2_CH_2_–OH, surrounding a polyether backbone that is chemically inactive, with terminal hydroxyl groups that can be triggered for conjugation to diverse types of polymers and drugs. Amphiphilic block copolymers like poloxamers and poloxamines, comprising hydrophilic PEG (or PEO), and hydrophobic PPO [poly(propylene oxide)] are additional forms of PEG products. These molecules are frequently employed for modification by surface adsorption or entrapment [91, 93]. The hydrophobic block of PPO anchors onto or entangles within the surface of hydrophobic nanoparticles matrices. The poloxamers are commercially available such as Pluronics from BASF Corporation that are *a*-*b*-*a* type triblock copolymers (PEO–PPO–PEO); poloxamines (or Tetronics) are tetrablock copolymers of PEO–PPO joined by an ethylenediamine bridge ((PEO–PPO)_2_–x–(PPO–PEO)_2_) [94–96]. The equilibrium among hydrophilic and lipophilic segment of these copolymers can be adjusted through variations of the molecular weight of “*a*” and “*b*” blocks. As an example, Pluronic F-108 NF, a poloxamer 338 molecule, has a bulkier middle block. It has longer side arms containing *a* = 122 and *b* = 56. These side arms can be compared to Pluronic F-68 NF, containing poloxamer 188 possessing longer side arms with *a* = 76 and *b* = 30. This dissimilarity can impart a significant modification property such as in the physicochemical properties of the triblock copolymer that control its applicability. An instance of surface modification helps in the variation of poloxamers. In this case, variation of *a* : *b* ratios is important and can be prejudiced for biodistribution of PCL nanoparticles. For example, it was observed that 74% of Pluronic F-68 NF and modified nanoparticles gather within the liver after 1 hour of administration. Whereas only 67% of Pluronic F-108 NF altered nanoparticles accumulated in the liver. Moreover, modified nanoparticles are less toxic compared to unmodified (83%) nanoparticles as PEG surface-shielding helps to avoid recognition by the RES system [97].

The article "Recent Trends of Polymer Mediated Liposomal Gene Delivery System" was retracted in 2019. Reasons: plagiarized text; overlap with other authors' work.

### 3.3. Polymeric Nanoparticles and PEG Chains

Surface modification of the polymeric nanoparticles can also be achieved through covalent bonding by grafting of PEG chains against the nanoparticle surface, and likewise through the use of copolymers, according to which PEG is covalently linked to another polymer type. However, PEG modification can also be achieved by noncovalent bonding of surface adsorption or entrapment into the nanoparticle matrix [91]. Some of examples regarding PEG modification by covalent and noncovalent bonding are presented elsewhere [98]. PEG offers an important advantage for the nontoxic and nonimmunogenic gene transfer which is internally used in humans. It proves the evidence for inactive ingredients for oral as well as parenteral applications which is approved by the USFDA [99]. An extensive range of molecular weights of PEG is available up to several million daltons (Da). It is not biodegradable and influences its elimination from the body. Yamaoka et al. [100] discovered that molecular weight of PEG up to 20 kDa is initially excreted through the renal system. Finally, the PEG chains show higher molecular weight transition from urinary to fecal excretion.

### 3.4. Molecular Weight, Size, Shape, and Other Parameters of PEG Chains and Application as Delivery System

Depending on the increase in variations of molecular weight, defined by the number of repeating units, PEG chains can be produced in two conformations, as either linear or branched chains [101]. The defensive performance of PEG is usually due to the development of thick, hydrophilic cloud of long flexible chains on the colloidal surface that reduces the hydrophobic interactions with the RES. The tethered and chemically anchored PEG chains can undergo spatial conformations. Consequently, it is avoiding the opsonization of particles via the macrophages of the RES and thus favors accumulation in liver and spleen. Therefore, PEG surface modification enriches the circulation time of the colloidal particles in the blood [92, 102, 103].

The article "Recent Trends of Polymer Mediated Liposomal Gene Delivery System" was retracted in 2019. Reasons: plagiarized text; overlap with other authors' work.

The method of steric hindrance by the PEG modified surface has been thoroughly inspected [93]. A structured shell is formed by the water molecules through hydrogen bonding to the ether oxygen molecules of PEG. The protein interactions are repelled by the strongly bound water that forms a hydrated film around the particle [104]. Additionally, PEG surface modification also increases the hydrodynamic size of the particle and reduces its clearance. This process is dependent on the molecular size as well as particle volume [105]. Eventually, these assistants are greatly increasing circulation half-life of the particles [91, 102, 106]. The technology of PEG modification is readily in use, for example many PEG-modified nanocarrier products have been developed for tumor targeting which have been noted elsewhere [98].

The molecular weight, size, and shape of the PEG segment and the kind of linkage used to connect it to the entity of interest define the significances of PEGylation in relation to protein adsorption and pharmacokinetic properties like volume distribution, circulation half-life, and renal clearance. The required amount of PEG on the colloidal surface can be adjusted by altering the molecular weight and molar ratio (e.g., grafting efficiency) of PEG integration, when formulated into colloidal particles. Longer PEG chains offer better steric influence around the colloidal entity and the related phenomenon have been seen when the grafting density is increased in regard to the PEG chain length. Longer PEG chains may also collapse against the nanoparticle surface to provide a hydrophilic shield [107]. But, steric-shielding enhances therapeutics circulation time. It is not astonishing that colloidal particles modified with 6.5 mol% PEG that usually have a longer circulation time (half-life of 170 min) than particles changed with 2.5 mol% PEG (half-life of 80 min).

Remarkably, branched derivatives of PEG usually have an increased half-life over unbranched PEG chains. But, at 7 or greater mol% surface modification, both unbranched and branched derivatives show a similar steric effect. There exist many reports to support the pharmacokinetic enhancements that have been observed with the use of PEG-modified nanocarriers over unmodified nanocarriers. For example, gelatin nanoparticles which are modified by PEG chains show increased circulating half-life from 3 to 15 h over unmodified gelatin nanoparticles, evidenced by a three-fold reduction in total body clearance [108]. Nanocarriers with prolonged circulation time and 29 to 38 h of half-life are considerably required to enrich tumor tissue, a significant enhancement of therapeutic efficacy. Likewise, a PLGA nanocarrier with PEG-modification also improves the circulation time. Only 5% of unchanged particles remains in circulation within 5 min of administration; nonetheless as much as 25% of PEG of molecular weight of 5 kDa continues circulation [103]. Remarkably, PLGA particles that had been modified with 20 kDa molecular weight of PEG were reserved up to 50% of the circulation within first 5 minutes. This observation supports the increasing stealth properties and decreasing clearance for longer PEG chains.

The article "Recent Trends of Polymer Mediated Liposomal Gene Delivery System" was retracted in 2019. Reasons: plagiarized text; overlap with other authors' work.

Some nanomaterials such as fractured dendrimer and polyethyleneimine were also used through* in vivo* study and are shown to be active in brain and carotid artery [109, 110]. The gene relocation by polyplexes and lipoplexes is less efficient* in vivo* than* in vitro*.* In vitro* effects are not predicted well in case of* in vivo* gene transfer [111, 112] because of the different biological barriers* in vivo*, factors that are not present* in vitro* cell culture systems. The complex formation of cationic vehicle and DNA may interact with the extracellular matrix materials after local gene administration (e.g., in arterial walls, vitreous of the eye, joints, dermis, extracellular matrix in tumor, etc.) and such communication may hinder the gene transfer to the targeted cells.

Extracellular matrices comprise sulfated proteoglycans that consist of a core protein covalently linked to one or more sulfated or carboxylic glycosaminoglycans (GAGs) [113]. Negatively charged GAGs, such as hyaluronic acid and chondroitin sulfates, are long unbranched polysaccharides with repeated sulphated or carboxylic disaccharide units [112, 113]. Extracellular polyanionic GAGs might bind the positively charged DNA complexes and, thus, disturb their mobility in tissue, as well as interaction with target cells.

Previously, Xu and Szoka [114] presented some polyanions (heparin and dextran sulfate) that release DNA from DOTAP liposome by binding to the cationic lipids. Various polyplexes and lipoplexes are complexed with DNA differently and also their mechanisms and efficiencies in gene transfer are not alike [52, 62, 115–117]. Consequently, it has been demonstrated that the interactions between various DNA complexes and GAGs are far from identical. Additionally, inhibitory effects on transfection of cells are not dependent on DNA release or its relaxation in the complex.

The article "Recent Trends of Polymer Mediated Liposomal Gene Delivery System" was retracted in 2019. Reasons: plagiarized text; overlap with other authors' work.

Nonviral gene delivery schemes, for instance, cationic liposomes [118] or synthetic gene carriers, such as poly-L-lysine (PLL) [119–121], can overcome immunogenicity produced by viral vectors* in vitro*. However,* in vivo* applications of such gene delivery schemes are greatly destitute due to poor biocompatibility and rapid degradation [122]. The Lipofectin protocol is also one of the best dependable tools in this category [123]; nevertheless it also associated with high cytotoxicity [121]. To overcome these problems, PLL has been modified by covalently attaching compounds, like tyrosinamide triantennary oligosaccharide [124], asialoglycoprotein [118, 125–127],* N*-glutarylphosphatidylethanolamine [128], transferrin [120, 129], fusogenic peptide [129], antibody [130], lactose [131, 132], or mannose [133], for the use as a gene delivery vector. The terplex gene delivery system, consisting of plasmid DNA, low density lipoprotein, and stearyl-PLL, has been reported to improve the transfection efficiency [134]. Wolfert et al. [135] and Kabanov et al. [136] developed the A-B type block polycations as carriers for oligonucleotide and gene delivery. For these carriers, one hydrophilic polymer region, for example, PEG, is combined with PLL. This block copolymer forms a complex with DNA, maintaining a low cytotoxicity comparable to the cation alone but with high solubility. It also increases the transfection efficiency in cells, for example, in 293 cells (human primary embryonal kidney cells). Such results are strongly motivating to develop a new series of polymer carriers, like methoxy PEG-grafted PLL (PEG-*g*-PLL) carriers, named comb-shaped PEG-*g*-PLL copolymers. Choi et al. [137] found that the comb-shaped polymer had a 5- to 30-fold increase in transfection efficiency compared to PLL on Hep G2 cells. They also found that plasmid DNA/PEG-*g*-PLL complexes enter the cells through an endocytosis mechanism.

## 4. Gene Delivery

### 4.1. Gene Delivery as a Whole

Cationic polymers play a crucial role for the development of gene transfer agents due to their extraordinarily good potential to condense DNA [138]. The polycation-induced DNA condensation is usually expected to be an entropy-driven process [139]. The complex formation of high *M*_*W*_ polycations with DNA is thermodynamically preferred over the complexation with low *M*_*W*_ cations. The change of the entropy during complex formation is much higher if new counterion of the DNA is large and releases a huge number of low *M*_*W*_ counterions. As a result, the development of liposome-based gene delivery systems uses polycations to condense the DNA. This polymer/DNA complex is encapsulated by a liposome formulation leading to a liposome entrapped polycation condensed DNA [140]. A comparable approach was to incorporate the polymer/DNA complexes in biodegradable nanospheres and microspheres for controlled release of the complex [141]. Lipid molecules are the conserved entities for the formation of liposome which has a head group and hydrophobic hydrocarbon tail regions, linked through a backbone linker of glycerol [142]. Cationic lipids generally interact with a positive charge through one or more amines which are present in the polar head group. The presence of positively charged amines enables binding with anions, for example, those seen in DNA. Thus, accumulations of energetic contribution by forces like Van der Waals and electrostatic binding lead to the creation of liposome and also partially dictate the shapes attained by them [43]. Due to the polyanionic nature of DNA, cationic and neutral lipids are usually used for gene delivery even if the application of anionic liposomes has been fairly limited to the delivery of additional therapeutic macromolecules [143].

The article "Recent Trends of Polymer Mediated Liposomal Gene Delivery System" was retracted in 2019. Reasons: plagiarized text; overlap with other authors' work.

A large amount of effort has been made to deliver complexes composed of nucleic acid and liposome to target cells, organs, and/or tissues accurately with different delivery system (Figure 1). Ligands (having affinity to cell surface receptors) are usually attached to PEG and then to the cationic or anionic carriers. Owing to shielding the positive charge of cationic complexes by means of PEG, the delivery to a specific cell surface receptor is accomplished. Nevertheless, gene expression is usually lower in the target cell than using the nonspecific delivery of the cationic complex. PEG is unable to “deshield” upon contact with the target cell surface although PEGylation shields the positive charge on cationic complexes. Therefore, the PEGylated complexes are not capable of utilizing critical charge interactions for optimal transfection into cells. This loss of positive charge on the surface causes transfection of fewer cells. First the half-life of complexes was increased by the use of PEGylation for the circulation and also to circumvent uptake in the lung. Conversely, this technology also abolishes the ability to transfect efficiently to the cells. The transfer of PEGylated complexes into cells occurs predominantly through the endocytic pathway. Subsequent deprivation of the DNA has been observed in lysosomes. It is considered that maintenance of sufficient positive charge on the surface of complexes is necessary to drive cell entry by direct fusion. Templeton [144] produced targeted delivery of the complexes without the use of PEG and even tried to maintain the overall positive charge. It was achieved either through ionic interactions or covalent attachments of Fab fragments, monoclonal antibodies, proteins, partial proteins, peptide mimetics, peptides, small molecules, and drugs to the surface of the complexes after mixing. These ligands obviously enhanced the entry of complexes into the cell either by direct fusion or by competently binding to the targeted cell surface receptors. Novel approaches of adding ligands to the complexes for targeted delivery may further increase the gene expression levels in the targeted cells after transfection. For this reason, Templeton [144] designed targeted liposomal delivery systems that could predominantly enter cells by direct fusion rather than endocytic pathway.

The article "Recent Trends of Polymer Mediated Liposomal Gene Delivery System" was retracted in 2019. Reasons: plagiarized text; overlap with other authors' work.

### 4.2. Gene Delivery through Liposome: Basis and Status

The reported lipid-polymer hybrid systems include DNA precondensed with polycations followed by coating with cationic liposomes [145, 146], anionic liposomes [147], or amphiphilic polymers with or without helper lipids [148]. Linear poly-L-lysine, protamine, histone, and various synthetic polypeptides have been used as the DNA condensation component; the polyplexes formed are then coated with a lipid layer. DNA is better protected in these lipid-wrapping polyplexes.* In vitro* [145, 146], the 3-part structure seems to be more efficient in transfection than lipid-DNA complexes and is true even for* in vivo* efficiency [149]. An extensive reorganization of the lipid membranes takes place following the initial contact when anionic complexes and DOPE-rich liposomes are added to DNA polycation complexes which results in lipid-polymer-DNA complexes with anionic lipid coatings [147]. This method overcomes the surface charge issue associated with cationic lipid-polymer-DNA complexes. The receptor-mediated targeting is made possible by reducing cytotoxicity of the complexes without interfering with nonspecific charge-charge interaction. A parallel approach also resulted in a functional complex that can be used for targeted gene delivery using amphipathic peptide derivatives as DNA packing agents and a bulk of neutral helper lipid to prepare DNA complexes by the detergent dialysis method [150]. Lately, numerous aspects related to lipid composition, the presence of shielding PEG-lipid conjugates, and the nature of chemical bonding that contributes to the biodegradability of the PEG-lipid conjugates in cells have been thoroughly studied [151, 152]. Such ideas are significantly not the same from the original lipid-DNA and/or polymer-DNA complexes and certainly deserve further exploration, particularly in the area of* in vivo* targeted gene delivery.

The article "Recent Trends of Polymer Mediated Liposomal Gene Delivery System" was retracted in 2019. Reasons: plagiarized text; overlap with other authors' work.

Human telomeric DNA is composed of typical thousands of TTAGGG repeats completed with 100–200 nucleotides at 3′-end overhang [153]. These DNA sequences* in vitro* can form four-stranded helical structures called G-quadruplexes, [154–157] assembled from the stacking of multiple G3G3G3G tetrads [158]. G-quadruplexes at telomeres have been noticed* in vivo* [159], and their presence in living cells can be regulated by a number of proteins [159, 160]. Intramolecular G-quadruplexes created by human telomeric DNA sequences are promising anticancer targets [161, 162], because the formation of such structures by the telomeric 3′-end overhang inhibits the activity of telomerase [163, 164], an enzyme essential for the proliferation of most human cancer cells [165]. Biological macromolecules in living cells function in a crowded intracellular environment [166–168]. Molecular crowding may perhaps affect the structure, stability, and activity of biomolecules [166–168]. Many groups used circular dichroism (CD) spectra to interpret structural alterations of G-quadruplexes under molecular crowding situations [169–175]. Miyoshi et al. [170] reported that molecular crowding simulated by PEG induces conformational development of an Oxytricha telomeric sequence from an antiparallel to a parallel-stranded G-quadruplex. Similarly, PEG was shown to induce conformational development in a human telomeric sequence [171, 174], and it has been recommended that 40% (w/v) PEG bring conformational switch of this sequence from an antiparallel to a parallel-stranded G-quadruplex [174]. Under some circumstance, such as under molecular crowding, the role of hydration on G-quadruplexes was discussed in the work of Miyoshi et al. [172], using different carbohydrate cosolutes, and of Vorlíčková et al. [173], using ethanol cosolute. A recent work by Miller et al. [176] showed that 50% (v/v) of acetonitrile could induce conformational development in a human telomeric sequence and hydration is necessary for determining the shape of G-quadruplex. However, the G-quadruplex conformation made in this condition [176] was not identical to the parallel form observed in the crystalline state [177]. Heddi and Phan [178] found that different G-quadruplex shape may change into a propeller-shaped G-quadruplex. Study reported conversion of four different G-quadruplex conformations to a propeller-type parallel-stranded G-quadruplex in potassium- (K^+^-) containing crowded solution, due to depletion of water. They also observed complex level of arrangement in extremely water-depleted condition, solutions containing high levels of PEG concentration.

The article "Recent Trends of Polymer Mediated Liposomal Gene Delivery System" was retracted in 2019. Reasons: plagiarized text; overlap with other authors' work.

Liang et al. [179] prepared cationic polymeric liposomes (CPLs), with lipid bilayer structure having high thermal stability provided by polymeric surfactants of quaternized (carboxymethyl) chitosan attached to different carbon chains (namely, dodecyl, tetradecyl, hexadecyl, and octadecyl). The gene delivery can be achieved through tetradecyl-quaternized (carboxymethyl) chitosan (TQCMC) CPLs, having a suitable size of about 184 nm, *ζ* potentials of about 27 mV, and productivity for synthesis of TQCMC with weight yield of 13.1%, in different cancer cell lines. It is resolved that the CPLs are favorable gene delivery schemes that might be used to target different cancers. The transfection of internalized polyplexes depends on the cell type and the kind of polymer used. It has been reported that the clathrin-coated pit pathway is the main route of transfection for linear polyethylenimine (PEI) polyplexes [180]. Branched PEI polyplexes appear to facilitate transfection via both the clathrin-dependent and lipid-raft-dependent pathways. However, both pathways are involved in HeLa cells, with the former being more pronounced [180]. In A549 and HeLa cells, [181] PEI polyplexes are internalized by both pathways, but polyplexes taken up by clathrin-mediated endocytosis are degraded in lysosomes, while those entering cells via caveolae are successful in transfection [181]. van der Aa et al. [182] showed that in COS-7 cells, blocking caveolae-mediated uptake causes an almost complete inhibition of PEI and pDMAEMA polyplex-mediated gene expression, while internalization proceeds by both the clathrin and caveolae-mediated pathways. However, the use of a specific inhibitor of fluid-phase endocytosis designated that this route is involved in internalization of PEI-25-DNA complexes and transfection in CHO-K1 and HeLa cells [183]. Hatakeyama et al. [184] recently found a multifunctional envelope-type nanodevice (MEND) to be used as a novel nonviral gene delivery system. The modification of PEG, that is, PEGylation, is an appropriate method for attaining a longer passage time for the transfer of MEND to a tumor through the improved permeability and retention (EPR) effect. PEGylation helps to strongly inhibit cellular uptake and endosomal escape which could otherwise result in significant loss of activity of the delivery system. This study described the developments and the applications of MEND and various strategies based on the control of both the pharmacokinetics and cell trafficking, basically intracellular trafficking during the cellular uptake process and endosomal discharge which occurred to overcome the PEG dilemma. In response to the intracellular environment and the tumor microenvironment, the separation of PEG from carriers was achieved to improve cellular uptake and endosomal escape.

The article "Recent Trends of Polymer Mediated Liposomal Gene Delivery System" was retracted in 2019. Reasons: plagiarized text; overlap with other authors' work.

## 5. Future Direction

The field gene therapy is making excellent progress. Many gene therapies are showing very significant result and are in clinical trials. Some instances of gene therapies are in the management of haemophilia B and lipoprotein lipase scarcity [185, 186]. However, there are some hazards associated with the polymer mediated liposomal gene delivery vectors and thus future researches focused on making safer gene delivery system are required. More advanced polymer mediated liposomal gene delivery vectors are required for site specific deliveries. So that, it can be utilized for specific diseases, through definite routes as well as for exact tissues. Still, some studies are needed to improve the efficacy of the polymer mediated liposomal gene delivery system for clinical applications. Parallel to this, a newer polymer mediated liposomal gene delivery system is required for reducing observed drug toxicities. Finally, a cost effective and cheaper gene therapy can help maximize not only the people from the developed countries but also the people from the developing world.

## 6. Conclusion

A wide variety of gene delivery systems has already been technologically advanced, and many such systems are in the growing phases for the therapy of genetic diseases [187]. It has been observed that the polymer structure has a strong effect on the shape of the lipid/DNA complexes. The transfection of polyplexes within the cell is influenced by the cell type and the kind of polymer used. Biological macromolecules in living cells, function in a crowded intracellular environment and such crowding, might affect the structure, stability, and activity of biomolecules. Cationic polymer plays a key role in the development of gene transfer agents because of their well-defined potential to condense DNA. Large and diffusive complexes with positive surface charge are made using polymers with many short PEG blocks. Such polymers, using a long PEG blocks, can self-assemble into small and compact condensates of lower surface charge. However, a high positive *ζ*-potential of the complexes can cause a robust erythrocyte aggregation and haemolysis. Cytotoxicity monitored with fibroblasts has a function of the degree of PEGylation independent of the molecular weight of the PEG. Appropriate* in vitro* gene expression is realized with the polymer that created large complexes with a large surface charge and a low toxicity profile, as it is found for the polymer with several PEG blocks.

The article "Recent Trends of Polymer Mediated Liposomal Gene Delivery System" was retracted in 2019. Reasons: plagiarized text; overlap with other authors' work.

## Figures and Tables

**Figure 1:** Structure of liposome and schematic representation of the polymer modified liposomal gene delivery; (a) structure of liposome and its different phases: (i) gel phase and (ii) liquid crystalline phase; (b) schematic representation of the polymer modified liposomal gene vehicle preparation and release process after the delivery in the cell.
